# Gravitational Wave-Signal Recognition Model Based on Fourier Transform and Convolutional Neural Network

**DOI:** 10.1155/2022/5892188

**Published:** 2022-09-29

**Authors:** Hao Zhang, Zhijun Zhu, Minglei Fu, Minchao Hu, Kezhen Rong, Dmytro Lande, Dmytro Manko, Zaher Mundher Yaseen

**Affiliations:** ^1^China Mobile Group Zhejiang Co., Ltd, Hangzhou 310006, China; ^2^College of Information Engineering, Zhejiang University of Technology, Hangzhou 310023, China; ^3^Institute for Information Recording, National Academy of Sciences of Ukraine, Kyiv 03113, Ukraine; ^4^Civil and Environmental Engineering Department, King Fahd University of Petroleum and Minerals, Dhahran 31261, Saudi Arabia

## Abstract

The recent detection of gravitational waves is a remarkable milestone in the history of astrophysics. With the further development of gravitational wave detection technology, traditional filter-matching methods no longer meet the needs of signal recognition. Thus, it is imperative that we develop new methods. In this study, we apply a gravitational wave signal recognition model based on Fourier transformation and a convolutional neural network (CNN). The gravitational wave time-domain signal is transformed into a 2D frequency-domain signal graph for feature recognition using a CNN model. Experimental results reveal that the frequency-domain signal graph provides a better feature description of the gravitational wave signal than that provided by the time-domain signal. Our method takes advantage of the CNN's convolution computation to improve the accuracy of signal recognition. The impact of the training set size and image filtering on the performance of the developed model is also evaluated. Additionally, the Resnet101 model, developed on the Baidu EasyDL platform, is adopted as a comparative model. Our average recognition accuracy performs approximately 4% better than the Resnet101 model. Based on the excellent performance of convolutional neural network in the field of image recognition, this paper studies the characteristics of gravitational wave signals and obtains a more appropriate recognition model after training and tuning, in order to achieve the purpose of automatic recognition of whether the signal data contain real gravitational wave signals.

## 1. Introduction

On September 14, 2015, the laser interferometer gravitational wave observatory (LIGO) achieved the first direct detection of gravitational waves in human history. Subsequently, gravitational wave detection developed rapidly. On August 14, 2017, two LIGO project teams in the United States and the Virgo team in Europe detected a new gravitational wave event nearly simultaneously using three separate gravitational wave detectors [1]. Because the event was detected by different machines and project groups, the detection results were rendered more authentic and credible [2]. On October 3, 2017, Rainer Weiss, Barry Clark Barish, and Kip Stephen Thorne won the Nobel Prize in physics for their contributions to the discovery of gravitational waves. Not surprisingly, the number of gravitational wave detection events has increased [3, 4].

The traditional gravitational wave detection method uses a matched filtering method [5]. This method has shown excellent performance in wave-signal extraction. However, matched filtering also has defects. First, the computation costs are huge, making the data-processing speed very slow. In addition, the premise of matched filtering is that an accurate theoretical template is needed. This can result in gravitational wave signals not being detected if they are beyond the theoretical expectation [6].

As an emerging field, deep learning (DL) has developed rapidly over the past decade and has attracted increasing attention from researchers [7–9]. With the increasing capabilities of computer hardware and the development of adaptive software, powerful feature extraction and generalization capabilities are now available [10–12]. Such machine-learning capabilities allow data to be processed at higher recognition rates and with better accuracy [13]. Notably, these advantageous DL methods have been applied to the data processing of gravitational wave detection. For example, to promote astronomical breakthroughs and accelerate the detection and analysis of gravitational wave signals, Bahaadini et al. [14] proposed a machine-learning method to distinguish clustering data and to classify and identify gravitational wave faults [15, 16]. George and Huerta [17] used depth filtering to detect gravitational wave signals and tested the feasibility of applying DL methods to signal recognition [18]. They also introduced a denoising autoencoder to improve recognition performance [19]. Since then, many scholars have developed new methods to optimize performance, including Li et al. [20] applied a Gaussian-noise technique to the wavelet decomposition of simulated gravitational wave signals to improve resolution accuracy. Fan et al. [21] used signal data from multiple sources to enhance the performance of neural networks for parameter estimation. Chua et al. [22] used a reduced-order modeling method to represent waveform data and derived a learning model built upon the Bayesian method [23]. Cao et al. [24] designed a new convolutional neural network structure, which only uses dozens of waveforms in the sensing layer and clearly identified 11 gravitational wave events that had been confirmed at the time. Gabbard et al. [25] constructed a deep convolutional neural network, which can reproduce the sensitivity of matched filtering method to search gravitational wave signals of binary black holes. Luo et al. [26] tracked and copied the code posted on GitHub by Gabbard et al. and found that, in their model, the fitting effect of the training set was much higher than the generalization effect of the test set, suggesting that there might be an over-fitting problem. They optimized the model to achieve better accuracy. Wei and Huerta [27] applied DL integrated system to detect gravitational waves from the merging of rotating black holes in real time. The reported literature provided several pathways for future combinations of DL and gravitational wave detection.

In summary, many teams have leveraged DL methods to successfully identify real gravitational wave signals [28, 29]. However, in the previous studies, the collected data were all applied to time-series signal processing, which would led the convergence in the training process to intractable, and the final detection accuracy is also not satisfactory. In other word, the main problems need to be settled contain how to get the datasets of Gravitational wave signals and the difficulties in designing models and training models:

- The signal of the training data is too strong to be matching, but too weak to be trained. Therefore, proper SNR classification of the data set is needed.
- The selection of the core size of convolution layer and pooling layer should conform to the characteristics of the input image.
- The number and layer of neurons is not the more the better; there is an optimal number and layer.
- The number and layer of neurons is not the more the better; there is an optimal number and layer. The selection of activation function and learning rate will affect the training speed and accuracy of the model. Hence, in this study, the proposition of the transformation of the time-domain signal of gravitational waves into 2D frequency-domain signal graphs for feature recognition was suggested. This is for the purpose to make full use of convolutional neural network (CNN) image processing and improve the overall recognition accuracy.

The remainder of the study is organized as follows. In Section 2, the gravitational waves and data collection are explained. Comprises the methods and materials used in our study. In Section 3, the experimental results are analyzed. Finally, Section 4 summarizes the attained results and discusses prospects.

## 2. Generation Principle of Gravitational Waves and Dataset Acquisition

### 2.1. Generation Principle of Gravitational Waves

According to general relativity, gravitational waves are naturally generated by several astrophysical phenomena [28, 30]. There are three main sources of gravitational waves [31]: the expanding and changing universe [32], continuous waves from rotating deformed neutron stars, and unmodeled burst signals from supernovas [33, 34]. Most of the observed gravitational wave events are produced by black-hole mergers. One such merger involved two revolving black holes having masses of 31 and 25 times the mass of the sun, *M*_*sun*_. After their merger, the mass of the new black hole was 53 *M*_*sun*_; the remaining 3 − *M*_*sun*_ mass was released in the form of gravitational wave energy.

### 2.2. Dataset Acquisition

Our team studied the gravitational waves formed by the merger [35]. The parameter space of the gravitational wave was sufficiently small to meet the needs of this study. Therefore, a gravitational wave radiated by the black-hole system without spin was considered [36]:

(1) $$\begin{array}{c} \begin{array}{c} h=F_{+}h_{+}+F_{\times }h_{\times } \end{array}\text{,} \end{array}$$

where *h*_+_ and *h*_×_ are the two polarization modes of the gravitational wave and *F*_+_ and *F*_×_ are the response functions of the detector to the two polarization modes, respectively. We assume that the detector was placed ideally, *F*_+_=1 and *F*_×_=0. In other words, only the “+” polarization mode of the gravitational wave is considered. An effective unit numerical relativistic model was used to simulate the gravitational wave signal.

In order to standardize the input data, reduce the adverse effects caused by the singular sample data, and thus reduce the accidental experiment, we normalized the gravitational wave shape and focused on its signal, which lasted for 1 s. It is the case that the most difficult to distinguish among gravitational waves are transient non-Gaussian noise signals called “glitches.” Zooniverse's gravity monitoring project has selected 22 different types of noise, with short-duration noise being the majority. In addition, according to the results obtained by Bahaadini et al. in [14], the `single-view model with shorter burrs has better class performance for shorter burrs. Finally, combined with the convenience of data processing in the frequency domain, the observation time of gravitational waves is determined to be 1 S. The sampling frequency of the gravitational wave data was 8,192 Hz, corresponding to 8,192 data points over 1 s. To study the influence of the signal-to-noise ratio (SNR) on the accuracy of data training, we preprocessed the data to obtain different SNRs for comparative training. Simultaneously, for the time-domain data, we carried out a discrete Fourier transform:

(2) $$\begin{array}{c} \begin{array}{c} X\left(e^{jw}\right)=\overset{+\infty }{\underset{n=-\infty }{\sum }}x\left(n\right)e^{-jwn}. \end{array} \end{array}$$

A converted frequency-domain data graph was obtained [37, 38]. As shown in Figures 1(a)–1(d), the gravitational wave mixed-noise waveforms (SNR = 8 and 2) and the gravitational wave mixed-noise spectrum (SNR = 8 and 2) are presented, respectively.

### 2.3. Data-Processing Method

As a classical application of deep learning, CNNs produce excellent results in the field of image recognition [39, 40]. A basic CNN consists of an input layer, a convolution layer, a pooling layer, a fully connected layer, and an output layer. The input layer processes multidimensional data. According to the input data type, a 1D, 2D, or 3D CNN can be selected. To improve its learning efficiency, the input data should be normalized. The convolution layer provides the core functionality, which can extract features from data. The efficiency of feature extraction depends on the CNN layer's convolution kernel. For different requirements, it is necessary to design an appropriate convolution kernel size. After feature extraction in the convolution layer, an output feature map is transmitted to the pooling layer for information selection and filtering. Following multiple convolution and pooling layers, the final extracted features enter the fully connected layer as a nonlinear combination to produce the output. The final layer outputs the data according to the pre-set classification criteria.

We used an Intel i7 processor with an eight-core processor. In the TensorFlow platform, the Keras library was called to train the model, and the Adadelta method was used in the gradient-descent optimizer.

Based on the powerful performance of CNNs, our team designed and experimented with relevant models regarding their application to gravitational wave recognition problems, as shown in Figure 2.

### 2.4. Time-Domain Model Training

We divided the dataset into signal + noise data and noise-only data. To balance the accuracy of the model and training speed, we analyzed and tested its structure and finally obtained a relatively good model (Figure 3).

The model consisted of three convolution layers and three pooling layers. The convolution layers were used to extract features. In the selection of activation functions, we consider the commonly used activation functions, including Sigmoid function, Tanh function, and ReLU function. However the first two functions both are evaluated using exponents, which lead to inefficiency. Therefore, the activation function used the rectified linear-unit (ReLU) function as

(3) $$\begin{array}{c} \begin{array}{c} f\left(x\right)=\max\;\left(0,x\right). \end{array} \end{array}$$

This function can effectively solve the problem of gradient vanishing and accelerate training speed. There was a pooling layer after each convolution layer, and maximum pooling was used. Finally, there was a fully connected layer, where the softmax function was used as the output of the second layer. The cross-entropy loss function is

(4) $$\begin{array}{c} \begin{array}{c} C=-\frac{1}{n}\underset{x}{\sum }\left[y\;\ln\;a+\left(1-y\right)\ln\;\left(1-a\right)\right], \end{array} \end{array}$$

where *a*=*σ*(*z*), and

(5) $$\begin{array}{c} \begin{array}{c} z=\sum w_{j}\cdot x_{j}+b, \end{array} \end{array}$$

where *C* is the loss function, *n* is the total number of samples, *x* is the sample, *a* is the actual output of the neuron, *y* is the expected output, *w*_*j*_ is the weight, *x*_*j*_ is the random variable, and *b* is the bias. The derivation of *C* was performed as follows:

(6) $$\begin{array}{c} \begin{array}{c} \frac{\partial C}{\partial w_{j}}=\frac{1}{n}\underset{x}{\sum }x_{j}\left(\sigma \left(z\right)-y\right)\text{,}\\ \frac{\partial C}{\partial b}=\frac{1}{n}\underset{x}{\sum }\left(\sigma \left(z\right)-y\right)\text{.} \end{array} \end{array}$$

It can be observed that the weight update was affected by the error. The larger the error, the faster the weight update.

Besides that, gradient descent algorithm is also important for neural networks. After two optimization improvements of SGD algorithm and Adagrad algorithm, Adadelta algorithm has made significant progress. On the basis of Adagrad algorithm, Adadelta algorithm introduces a new “dynamic learning rate” to reduce the repetitive task of repeatedly selecting the learning rate and does not need to manually set the learning rate, reduces the amount of calculation, and has good robustness for large gradient, noise, and different structures. After the approximate Newtonian iteration, the expression could be written as follows:

(7) $$\begin{array}{c} \begin{array}{c} ∆\theta_{t}=-\frac{\sqrt{\sum_{t=1}^{t-1}∆\theta_{t}}}{\sqrt{E\left|g_{t}^{2}\right|+\varepsilon }} \end{array}\text{,} \end{array}$$

where *g*_*t*_ is gradient, *E* is the value of expectation, ∆*θ*_*t*_ represents the learning rate, *ε* is the constraint, and *t* is the iterations. At this point, Adadelta algorithm no longer relies on the global learning rate, but uses exponential decay moving average to discard distant historical information. Its characteristics are, in the early and middle training, the acceleration effect is faster, and in the late training period, the local minimum was jitter repeatedly. And combined with the special characteristics of gravitational wave spectrum recognition, we choose Adadelta algorithm as the gradient descent algorithm of neural network.

The data then in the training set were used to train the model for 200 epochs. We found in the experiment that, in the frequency domain, the loss had dropped to close to zero in the 100th iteration, and in the time domain, the loss function did not show significant fluctuations until close to 200 iterations. Each SNR was classified for training and testing. During each training epoch, there were 100 sets of training data. After several training sessions, the average accuracy was considered as the final accuracy under the SNR.

### 2.5. Frequency-Domain Model Training

Based on the time-domain model method, our team proposed a 2D image-input method to transform the time-domain data into a frequency-domain signal data graph using a fast Fourier transform. This method is more suitable for the excellent performance of CNNs for image recognition and processing. We fine-tuned the frequency-domain CNN model, as shown in Figure 4.

To adapt to the characteristics of the frequency-domain images, the number of model layers was not changed. However, the convolution kernel size was changed to 5 × 5. The same 200 cycles were used for training. The other processes were consistent with the time-domain data training. As shown in Figure 5, during the training process, the convergence speed of the frequency-domain model was slightly slower than that of the time-domain model, but it eventually converged. This supports the notion that the feature extraction effect of the frequency-domain data is better. The training time of the frequency-domain model was only half that of the time-domain model. Thus, the frequency-domain model had higher efficiency.

## 3. Experimental Results and Analysis

### 3.1. Comparative Analysis of Time and Frequency Domains

In order to comprehensively evaluate the performance of the design model, this study will change the image signal-to-noise ratio, the number of training sets, whether to carry out image filtering, using different models and other four aspects to carry out experiments while keeping other conditions unchanged. Accuracy and Error rate are the most critical evaluation indexes for binary classifiers. Acc and ERR are, respectively, listed:

(8) $$\begin{array}{c} \begin{array}{c} acc=\frac{TP+TN}{TP+TN+FP+FN}\text{,}\\ err=\frac{FP+FN}{TP+TN+FP+FN}\text{,} \end{array} \end{array}$$

where TP represents the number of positive classes predicted, TN represents the number of negative classes predicted, FP represents the number of positive classes predicted, and FN represents the number of negative classes predicted. TP + TN represents the number of correctly predicted samples, FP + FN represents the number of incorrectly predicted samples, and TP + TN + FP + FN represents the total number of samples. For binary classifiers, true and false are mutually exclusive events, so the sum of accuracy and error rate is 1. Therefore, this study selects accuracy rate as the final evaluation index of neural network to analyze its performance.

After several rounds of training and testing, the time-frequency comparison diagram shown in Figure 6(a) was obtained. The blue line represents the average correct rate of the time-domain test-set data under different SNRs. When the SNR was less than six, the accuracy rate dropped below 70% and decreased rapidly with the decrease in SNR. The accuracy of the frequency-domain data, represented by the red line, shows that the accuracy decreased slowly with a decrease in SNR. There still was approximately 70% accuracy when SNR = 2. When SNR = 11, the correct rates of the time and frequency domains were greater than 90%, indicating that both could be well resolved at high SNRs. However, with decrease in SNR, the characteristics of the gravitational wave in the time-domain data were not apparent and were dominated by noise, whereas the characteristics of the gravitational wave in the frequency-domain data could still be better learned and distinguished via machine learning. In summary, under the same noise interference, the gravitational wave characteristics of the frequency-domain data were more prominent, and the recognition effect was better than that of the time-domain data.

Figure 6(b) presents a comparison of matched and depth filtering fabricated by George and Huerta [2]. As can be seen from the figure, at low SNRs, the method did not recognize the wave. However, our frequency-domain method was effective. At higher SNRs, the two methods produce nearly the same results.

### 3.2. Research on Performance of the Frequency-Domain Model

The above experiments showed that the method of frequency-domain conversion of gravitational wave data containing noise could improve CNN recognition accuracy. Thus, to explore whether the performance of the selected model can be further improved, we conducted an exploratory experiment.

### 3.3. Image Filtering and Noise Reduction

The frequency-domain image of the gravitational wave signal was filtered using a mean filter:

(9) $$\begin{array}{c} \begin{array}{c} g\left(x,y\right)=\frac{1}{m}\sum f\left(x,y\right)\text{,} \end{array} \end{array}$$

where *m* is the total number of pixels, including the current pixel in the template. The filtered spectrum was used for training. As shown in Figures 7(a)–7(d), for different values (SNR = 8, 6, 4, and 2, respectively), the results obtained before and after the filtering algorithm were compared. The results revealed that, after using the filter, the accuracy of the training results were greatly improved when the number of training sets was small. With an increase in training sets, the accuracy of the test sets was slightly improved. Therefore, we can assume that the accuracy of the test set can be improved by filtering the frequency-domain image of the gravitational wave signal. In this study, we only used a simple filtering method for testing. In the future, we plan to obtain a better filter-preprocessing method to improve the effect of DL on gravitational wave signal recognition.

#### 3.3.1. Training-Set Increase

We selected data having SNRs of 8, 6, 4, and 2 for training and testing (as shown in Figure 8). The results demonstrate that increasing the training-set data increased the accuracy of the test set. When the training-set data increase from 100 to 400 groups, the average accuracy of the four groups increases by approximately 5%. However, owing to the extended training time, the impact of continuous improvement of training-set data on the overall accuracy almost disappears. Moreover, the consumption of computing resources increases significantly. Therefore, within a certain range, although the increase in the training set increases the training time, the test accuracy is significantly improved. However, beyond a certain range, the increase in training-set data has little impact on accuracy; however, it vastly increases time consumption.

### 3.4. Comparison of Deep Learning Models

To better illustrate the feasibility of the frequency-domain gravitational wave signal recognition method, we used the EasyDL platform developed by Baidu [41]. The existing mature Resnet101 model was used for verification training (Figure 9). As shown in Figure 9, under different SNR, the detection accuracy gap is about 6.5% when SNR = 2. The accuracy difference was about 2.5% when SNR = 10, and the final average accuracy difference was about 4%. Therefore, the results show that the recognition accuracy of the proposed neural network is about 4% higher than that of the third-party evaluation model. It proves that the scheme designed in this study has full rationality, feasibility, and superiority.

## 4. Conclusions

In recent years, several teams have applied DL methods to gravitational wave signal recognition, resulting in many published works. Most of these studies, however, applied time-series signal processes to discern gravitational wave signals. We proposed the first method to transform the time-domain signal of a gravitational wave into a frequency-domain signal via a discrete Fourier transform. This method helps extract the characteristics of the gravitational wave signal when using a CNN. We designed two CNN models for this purpose and tested their accuracies under multiple SNRs. Experimental analyses showed that the accuracy of recognition was improved by converting the gravitational wave signal to the frequency domain. After demonstrating the feasibility of this method, we designed several comparative experiments. Image filtering and training sets were used to enhance the recognition ability of the model. When the experimental results of the mature ResNet101 model were compared with those of the proposed model, it was observed that the proposed model achieved superior performance and surpassed our objectives. In future works, we hope to overcome current deficiencies and build a more efficient DL model. Furthermore, we hope to provide a better image-enhancement algorithm for preprocessing so that the model can better extract features and improve recognition accuracy.

## Figures and Tables

**Figure 1:** Gravitational wave mixed-noise waveforms: (a) SNR = 8 and (b) SNR = 2; gravitational wave mixed-noise spectra: (c) SNR = 8 and (d) SNR = 2.

**Figure 2:** Block diagram of detection system: (a) previous method and (b) our method.

**Figure 3:** Time-domain CNN model.

**Figure 4:** Frequency-domain CNN model diagram.

**Figure 5:** Comparison of loss values during the training process in time and frequency domains with SNR = 9.

**Figure 6:** Comparison with advanced detection network: (a) comparison of time- and frequency-domain accuracies with SNR variation and (b) sensitivity of detection with real LIGO noise [2].

**Figure 7:** Filter-contrast chart: (a) SNR = 8, (b) SNR = 6, (c) SNR = 4, and (d) SNR = 2.

**Figure 8:** Influence of increase in training-set data on test-set accuracy.

**Figure 9:** ResNet101 validation comparison.

## Data Availability

The data can be obtained from the corresponding author upon request.
